This article has been retracted.

# Modification in Silver Staining Procedure for Enhanced Protein Staining

**DOI:** 10.1155/2022/6243971

**Published:** 2022-05-13

**Authors:** Yibo Jiang, LinLin Zheng, Lulin Lin, Shan Lin, Kui Xu, SiJie Deng, QiQing Zhang

**Affiliations:** Department of Biomedical Engineering, Shenzhen People's Hospital (The Second Clinical Medical College, Jinan University, The First Affiliated Hospital, Southern University of Science and Technology), Shenzhen, 518020 Guangdong, China

## Abstract

Silver staining is an excellent technique for detecting proteins that are separated by sodium dodecyl sulfate-polyacrylamide gel electrophoresis (SDS-PAGE). Protein silver staining technology has higher sensitivity and is suitable for the detection of low-concentration proteins compared to other staining techniques including the Coomassie brilliant blue detection method. The present study was conducted to enhance the detection ability of the protein staining method. Herein, we modified the recipe of silver staining, a very reproducible method, by adding AMP, PVP, Tween-80, and xylene to enhance the detection ability of protein staining. Furthermore, the particle size and potentiometer were used to detect the particle size and potential difference of the silver ions in the prepared dyeing materials, and then, the morphology, transparency, and size of the dyed silver particles in different dyeing solutions were studied using a transmission electron microscopy (TEM). The obtained results revealed that the use of 0.5% of AMP, PVP, Tween-80, and xylene improved the staining ability of protein silver staining, compared with the original method. Furthermore, 0.5% AMP, 0.5% PVP, 0.5% Tween-80 reagents significantly influenced the morphology, size, potential, and dispersion of silver ions. These results suggested a new idea for further improving the detection ability of protein silver staining.

## 1. Introduction

Silver staining is an excellent technique for detecting proteins that are separated by sodium dodecyl sulfate-polyacrylamide gel electrophoresis (SDS-PAGE) due to its efficiency in detecting proteins present in nanograms. Protein silver staining is a nonspecific staining of proteins with an “explosive” reaction mode. This technique rapidly gained popularity owing to its high sensitivity as compared to other stains including the Coomassie Brilliant Blue R250 stains. The detection sensitivity was significantly enhanced by 20–200 times, allowing proteins as low as 0.1 ng protein per band to be detected [1, 2].

The technique is based on the simple principle that selective reduction of silver into metallic silver occurs at the initiation site in the proximity of protein molecules. The staining process sequentially consists of protein fixation, sensitization, washing, silver impregnation, and finally development of the image. Depending upon the amount of silver incorporated into the protein bands, a different color of the gel is produced on silver staining. Main SDS-PAGE and silver staining technique step are shown in Figure 1. Silver-stained protein bands generally are dark brown or black with considerable variation in color intensity. The color variation has been attributed to diffractive scattering by silver grains of different sizes. Few studies, however, demonstrated that color variation is due to the formation of silver chromate deposits that are incorporated into formalin-fixed proteins. It is also believed that the silver staining of protein bands is based on the combination of various groups in the protein (such as thiol and carbon group) with silver, resulting in the adhesion of silver ions to the surface of the protein, forming silver ion deposition, and encountering reducing agents that result in the precipitation of the color. The visualization of protein bands appeared as spots at the site of reduction, and therefore, the image of protein distribution within the gel is based on the difference in oxidation-reduction potential between the free adjacent sites and gel area occupied by the proteins. Numerous modifications to the silver staining procedure can alter the oxidation-reduction equilibrium, resulting in the visual representation of gel-separated proteins as positively or negatively stained bands [3]. However, proteins that do not contain or rarely contain cysteine residues are sometimes negatively stained [4, 5]. At present, the influence of the high-level structure of the protein on the silver staining effect cannot be determined.

Several factors influence the efficiency and sensitivity of silver staining. The concentration of the silver nitrate staining solution is determined by the gel thickness. For a gel with a thickness of 0.5–3 mm, a 0.1% concentration of silver nitrate is ideal, and larger concentrations should be utilized for ultrathin gels to compensate for diffusion through thin gels during formation. Aside from silver ions attached to proteins, silver ions in the vicinity of the protein are also required for the formation of bands. Another element that influences the sensitivity of protein staining on gels is protein reactivity with silver ions. The presence of amino acid in protein structure affects the process of silver staining. Staining was observed for the various homopolymers including polymethionine, the hydrophilic basic amino acid polymers: polylysine, polyarginine, polyornithine, and polyhistidine, [6]. Heukeshoven and Dernick also evaluated the silver staining of the basic homopolymers of arginine, histidine, and ornithine but not for polylysine [7]. According to Nielsen and Brown's observation, the basic amino acids lysine, arginine, and histidine, in both free orand homopolymeric forms, form colored complexes with silver reinforcing the role of the basic amino acids in silver staining [8]. The significant correlation between the intensity of silver staining and the mole percentage of basic amino acids lysine and histidine in a protein is most likely due to the electron-donating abilities of the amino groups and imidazole groups at the termini of the lysine and histidine side chains. At the termini of amino acid side chains, the amino and imidizole groups are capable of cooperating intramolecularly to bind silver ions, whereas the peptide bonding and N-terminal amino groups are not [3]. Histidine was found to be the most significant amino acid for silver ion binding and efficient silver staining among all amino acids. The histidine ligands connected the silver ions by binding through the imidazole nitrogen atom on one hand, and the N atom of the NH_2_ group on the other [9]. The reactivity of silver ions, and hence the sensitivity of protein detection, is also affected by protein structure. The functional groups of proteins must be exposed in order for silver ions to attach to them. As a result, native proteins are more reactive in silver staining than unfolded proteins produced by SDS.

However, when the technique was first established, it had various drawbacks, the most notable of which were a high background and frequent silver mirrors, as well as diminished sensitivity and reproducibility. To address these limitations, various changes were suggested from time to time, and hundreds of modified techniques for silver staining proteins on polyacrylamide gels are currently in use. We compared various modifications to the protocol of silver staining and examined the vital reaction steps and the effects of various additives to fixation solutions, such as glutaraldehyde and formaldehyde, and to the solution of silver staining, such as oxidizing agents [3], copper salts [10, 11], ammonium nitrate [12], and NaOH. In nearly all cases, adding these components to fixation, silver salt, or development solutions did not result in a well-defined enhancement of stained protein bands. Frequently, the additives resulted in an intensification of background staining. Such observations have led us to develop a more versatile silver staining protocol that requires only a few stable and readily storable solutions and allows for some coordinates in terms of concentration and reaction time.

In this study, we used 0.5% of AMP, PVP, Tween-80, and xylene which led to the enhancement of the silver staining technique. In addition, the particle sizer and the potential analysis system analyzed the potential and particle size of the silver dye reagent and the size, as well as the morphology of the silver dye particles. The morphology and structure of the silver particles in the silver dye reagent were observed and verified by TEM transmission electron microscopy technology. This study found that the morphological structure of silver particles is of great significance to the effect of protein silver staining technology and improving the sensitivity of silver staining. Relevant technical principles and methods provide a reference for further improving the detection effect and ideas of silver staining technology.

## 2. Methods

### 2.1. Gel Electrophoresis

The SDS-PAGE classic electrophoresis method was performed using the Beijing Liuyi electrophoresis instrument. Herein, we used commercially available BSA (bovine serum albumin) (Sigma fatty acid-free type) standard protein samples. The concentration and separation gels were 5% and 10%, respectively, with voltages of 80 V and 140 V. A 5X commercial SDS buffer (Tris-HCL PH6.8, 60 mM; SDS 2%; bromophenol blue 0.1%; glycerol 25%; *β*-mercaptoethanol 14.4 mM) was used. All reagents were made with premium-grade, which were mixed and boiled for 5 minutes before sample loading and electrophoresis. Following electrophoresis, a full piece of gel was obtained; however, during staining, the gel was separated and stained separately. A two-color 25-250KD protein marker was used as an electrophoresis label, followed by the gel documentation using the iBright Imaging System [1]. 2007, An et al. 2009).

### 2.2. Modified Method for Silver Staining

The gel was fixed with fixative solutions, i.e., ethanol (50%), glacial acetic acid (10%), and double-distilled water (40%) for 30 minutes, followed by gel treatment with ethanol (30%), sodium acetate (6.8%), and glutaraldehyde (0.6%) for 40 min. Next, 0.5% PVP (polyvinylpyrrolidone, molecular weight 58KD), 0.5% AMP (2-amino-2-methyl-propanol), and 0.5% Tween-80 were added, followed by adding 7.5% ethanol, 1.7% sodium acetate, 0.125% glutaraldehyde, and 0.2% sodium thiosulfate pentaerythritol and then soaked for 30 minutes. The gel washing was carried out in double-distilled water for 5 min, and then, silver staining was performed by adding 0.1% silver nitrate, 20% formaldehyde, and 0.5% xylene for 20 minutes, followed by adding 2.5% sodium carbonate and 10% formaldehyde for color development (10 minutes). The reaction was then stopped by adding 2% duodenum edetate for 10 minutes, followed by adding double-distilled water for washing thricely (5 minutes each time). According to the glue observation, the proper amount of double distilled water was added to save the gel.

### 2.3. The Measurement of Particle Size and Potential Difference

The particle size and potential difference were measured using a Malvern particle size potentiometer (ZEN 3700). First, 2 ml of the solution was added at 25°C temperature and the measurements were performed thricely. The average value was then used as the criterion after 10 minutes of stable measurements [13–15].

### 2.4. TEM Analysis

The morphology and structure of the silver particles in the silver dye reagent were observed and verified by TEM. First, eight samples (A-H) of silver ion materials were prepared including (A) 0.5% AgNO_3,_ (B) 0.5% AgNO_3_,0.5% Tween-80, (C) 0.5% AgNO_3_, 0.5% Tween-80, 0.5% AMP, (D) 0.5% AgNO_3_, 0.5% Tween-80,0.5% PVP, (E) 0.5% AgNO_3_, 0.5% AMP, 0.5% PVP, (F) 0.5% AgNO_3_, 0.5% PVP, (G) 0.5% AgNO_3_, 0.5% AMP, (H) and 0.5% AgNO_3_, 0.5% AMP, 0.5% Tween-80, 0.5% PVP. The samples were then subjected to ultrasonication for 10 minutes [16].

TEM (FEI Tecnai G2 Spirit Twin, Czech Republic) was used to observe the size and morphology of silver particles in various prepared solutions. Silurian materials were dyed with 2% phosphotungstic acid [17], and then, 10 *μ*L of the sample was dropped on a clean parafilm. The copper mesh upside was put down on the sample and suspended for 1.5 minutes. The copper mesh and filter paper were clamped and sucked up the excess liquid. Then, 10 *μ*L of 2% phosphotungstic acid was dropped on the clean sealing film. The dye solution on the copper mesh was suspended for 2.5 minutes. The copper mesh was clamped, and the excess liquid was absorbed with filter paper. All the consumables were dry at room temperature for 20 minutes. Tecnai G2 Spirit TEM was used for the photo of silver ion materials and the particle scale was calibrated at 500 nm at 4°C [15, 18].

Next, an image scale recognition software Image J (https://imagej.nih.gov/ij/) was used to perform image recognition and statistics of particle size. The statistical software SAS 12.0 was used to calculate the average value for each group. The significant level dividing line was *α* = 0.05 or 0.01 [13].

## 3. Results

### 3.1. Comparison of Dyeing Effects

We modified the traditional staining method by adding AMP, PVP, Tween-80, and xylene to enhance the detection ability of protein staining. As such, traditional staining methods have a poor effect, and the background remains high, resulting in limited detection capabilities for low-abundance proteins. The obtained results suggested that our recipe for protein silver staining makes the glue block more transparent and improves the overall yellow condition of the glue block. The combination of PVP, AMP, and Tween-80 kits resulted in more stained protein bands. Furthermore, the detection limit was estimated to be lower than 0.5 ng per protein band. In Figure 2(b), the bands from left to right are different concentrations of BSA protein, i.e., 20 ng, 50 ng, and 100 ng, and protein marker lysate. The image on the left is the result of the original method before optimization, and the image on the right is the result of the method after optimization. The result of the same batch of detection has a lower background and clearer bands.

Figure 3 shows the detection of BSA protein using electrophoretic staining. The electrophoresis bands in this experiment are BSA protein (20 ng, 50 ng, and 100 ng) and protein marker, from left to right.  Figure 3(a) shows the results obtained using the original untreated approach, while Figure 3(b) shows the results using the modified procedure with PVP, AMP, and Tween-80. Moreover, Figure 3(c) shows the results obtained from the new method, employed with PVP, AMP, and Tween-80, followed by treatment with xylene.

A comparative evaluation of the effects of various additives has been carried out. The quantitative findings of ultratrace BSA protein in an embodiment of the present invention are shown in Figure 4. Except for the marker, the protein concentration of the band from left to right was 0.1 ng, 0.2 ng, 0.5 ng, and 10 ng. The left picture is the original treatment group, the middle picture is the xylene treatment group, and the right picture is the posttreatment group with xylene. PVP, AMP, and Tween-80 were then added.  Figure 4(b) is whiter than the gel block on the right (Figure 4(c)), and the band with a protein concentration of 0.5 ng in the black arrow on the right is the most obvious, and the color rendering effect is significantly improved. The above-obtained results suggested that the new and improved method can effectively reduce the color rendering background, increase the color rendering brightness of the band, and improve the detection sensitivity.

The obtained results shown in Figure 5 demonstrate that adding reagents to the staining solution alone can boost the staining effect for a low concentration of the protein band. A protein concentration of 0.5 ng in the black arrow also has been shown. Compared with the original method, the sensitivity was improved after adding additives. Although the staining effect has been improved, the underlying explanation is still unknown.

### 3.2. Particles Sizes and Potential Analysis

Figure 6 shows considerable discrepancies between samples 1 and 2-8, as determined by the particle size potential analyzer ZEN 3700. The obtained results demonstrated that the smaller the potential, the larger the particle size. When compared to the standard reference group, each treatment group had a greater particle size and a lower potential. Among them, the composite treatment group 6 has the largest particle size and lower potential. Other reagents can increase particle size to varying degrees. This is sufficient to demonstrate that PVP, AMP, and Tween-80 decrease the silver ion potential and increase the particle size, which makes it easier for the particles to aggregate on the protein surface as an alteration in ion potential significantly affects the process of silver staining [6].

### 3.3. TEM Analyses

TEM analyses revealed that silver ion particles in samples 2–8 all get larger and more irregular in shape to varying degrees compared to sample 1(control) in Figure 7. It has been observed that the larger particles are more irregular in shape, as shown in Figure 7. Large particles are often between 200 and 300 nm in size but can reach 300 nm, while small particles are typically less than 100 nm in size. This result shows that treatment with PVP, AMP, and Tween-80 can increase the size of silver particles, facilitating the precipitation of silver ion particles on a large scale. Furthermore, the images also demonstrated the black spot which may be associated with the larger particle size of silver [3].

### 3.4. The Size of Each of the 100 Particles

According to the obtained statistics results, PVP and AMP treatment increases the size of AgNO_3_ particles to varying degrees. Although the exact cause of the final staining effect is complicated and dependent on several factors, this experiment reveals that using these reagents increases the size of the silver ion particles, as shown in Figure 8.

## 4. Discussion

Silver staining is an effective approach for detecting proteins separated by SDS-PAGE because of its efficiency in detecting proteins present in nanograms. It can be performed with simple and inexpensive laboratory reagents, and the readout does not necessitate complicated and expensive equipment.

Silver staining is the colorimetric approach that detects total protein with the highest sensitivity. Metallic silver is deposited onto a gel's surface at the positions of protein bands in this approach. Certain protein functional groups interact and bind with silver ions (from silver nitrate in the staining reagent). The most powerful interactions occur with carboxylic acid groups (Asp and Glu), imidazoles (His), sulfhydryls (Cys), and amines (Lys). Controlling the specificity and effectiveness of silver ion binding to proteins, as well as the successful conversion (development) of bound silver to metallic silver, necessitates the use of a variety of sensitizer and enhancer chemicals which can cause chemical crosslinking of the proteins in the gel matrix, limiting compatibility with destaining and elution methods for analysis by mass spectrometry (MS). The development process is nearly identical to that of the photographic film: silver ions are converted to metallic silver, yielding a brown-black color [18, 19].

Moreover, the unclear and high background makes it difficult to detect low-concentration proteins [8]. Hence, the present study conducted a new modified method for silver-stained polyacrylamide gel in protein staining, which can solve the problems of high background and insufficient color development in the existing silver staining.

Herein, an appropriate amount of PVP, AMP, Tween-80, and xylene was added during the staining to advance the sensitivity of silver stain detection and reduce the staining background which may result in the improvement of the target fragment brightness and the silver staining effect. The advanced phenomenon can result in the enhanced detection efficiency and sensitivity of low-concentration proteins.

Furthermore, the size of silver particles deposited on the protein surface has a significant impact on the protein gel's color development. In previous studies, it has been revealed that a reducing agent or the concentration of silver ions modulated the size of the silver ion particles. The potential difference when the particles aggregate can also affect silver ion aggregation [20]. In this study, the TEM results revealed that the larger the silver ion particles, the more irregular the shape, allowing for particles deposition. Hence, if large amounts of silver ions are deposited on the protein bands, it makes it easier to detect low-abundance proteins. PVP, AMP, Tween-80, and other reagents were used in this investigation to possibly influence the potential difference of silver ion particles, making it simpler for silver ion particles to form large particle deposits on the protein surface. Although the electric potential may not explain all the phenomena, it still reflects a certain trend for size of particles. The procedure described above resulted in an increase in detection sensitivity. As a result, the size of the potential plays a major role in particle and silver ion deposition on the protein surface, ultimately affecting the outcome of silver staining.

## 5. Conclusion

In this study, it has been revealed that the staining ability of protein silver stain was increased by adding 0.5% of AMP, PVP, Tween-80, and xylene. Furthermore, the background staining was decreased, which led to the enhanced detection efficiency and sensitivity of low-concentration proteins. PVP, AMP, Tween-80 also has an effect on silver ion shape, size, potential, and dispersion. This work presents a new approach to further enhance the protein silver staining detection technique.

## Figures and Tables

**Figure 1:** Modified method of silver staining.

**Figure 2:** SDS-PAGE of serial dilutions of BSA protein. (a) Staining according to the traditional method, and (b) staining with the new method.

**Figure 3:** Detection of BSA protein using electrophoretic staining (a) Original treatment method without xylene. (b) Treatment with PVP, AMP, and Tween-80 without xylene. (c) Treatment with PVP, AMP, and Tween-80 with xylene.

**Figure 4:** Comparison of the effects of various additives. The black arrow is 0.5 ng target protein. Target protein can be checked in both of B and C groups. (a) Original treatment group. (b) Xylene treatment group. (c) Xylene, PVP, AMP, and Tween-80 added group.

**Figure 5:** The black arrow is 0.5 ng target protein which is difficult to distinguish in (b) and even cannot be seen in (a). It is almost close to the limit of resolution. (a) Original method without other reagents. (b) The original method with the AMP group. (c) The original method with the Tween-80 groups.

**Figure 6:** The particle potential analysis: (a) 0.5% AgNO3; (b) 0.5% AgNO3 and 0.5% Tween-80; (c) 0.5% AgNO3, 0.5% Tween-80, and 0.5% AMP; (d) 0.5% AgNO3, 0.5% Tween-80, and 0.5% PVP; (e) 0.5% AgNO3, 0.5% AMP, and 0.5% PVP; (f) 0.5% AgNO3 and 0.5% PVP; (g) 0.5% AgNO3 and 0.5% AMP; (h) 0.5% AgNO3, 0.5% AMP, 0.5% Tween-80, and 0.5% PVP.

**Figure 7:** Eight samples (a–h) of silver ion materials: (a) 0.5% AgNO_3_; (b) 0.5% AgNO_3_ and 0.5% Tween-80; (c) 0.5% AgNO_3_, 0.5% Tween-80, and 0.5% AMP; (d) 0.5% AgNO_3_, 0.5% Tween-80, and 0.5% PVP; (e) 0.5% AgNO_3_, 0.5% AMP, and 0.5% PVP; (f) 0.5% AgNO_3_ and 0.5% PVP; (g) 0.5% AgNO_3_ and 0.5% AMP; and (h) 0.5% AgNO_3_, 0.5% AMP, 0.5% Tween-80, and 0.5% PVP. Ultrasonic treatment for each sample was for 10 minutes. The size and morphology of silver particles in various samples were observed. TEM was used to observe the size and morphology of silver particles in various prepared solutions.

**Figure 8:** The size of each of the 100 particles in samples (a–h): (a) 0.5% AgNO_3_; (b) 0.5% AgNO_3_ and 0.5% Tween-80; (c) 0.5% AgNO_3_, 0.5% Tween-80, and 0.5% AMP; (d) 0.5% AgNO_3_, 0.5% Tween-80, and 0.5% PVP; (e) 0.5% AgNO_3_, 0.5% AMP, and 0.5% PVP; (f) 0.5% AgNO_3_ and 0.5% PVP; (g) 0.5% AgNO_3_ and 0.5% AMP; and (h) 0.5% AgNO_3_, 0.5% AMP, 0.5% Tween-80, and 0.5% PVP. Each of the 100 particles was calculated on the basis of particle size.

## Data Availability

Data will be provided on request.

## Acronyms

TEM: Transmission electron microscope
NM: Nanometre
PVP: Polyvinyl pyrrolidone
AMP: 2-Amino-2-methyl-1-propanol.

## References

[1] Abdul-Rahman P. S., Lim B. K., Hashim O. H. (2007). Expression of high-abundance proteins in sera of patients with endometrial and cervical cancers: analysis using 2-DE with silver staining and lectin detection methods. *Electrophoresis*.

[2] Chevallet M., Luche S., Rabilloud T. (2006). Silver staining of proteins in polyacrylamide gels. *Nature Protocols*.

[3] Merril C. R. (1986). Development and mechanisms of silver stains for electrophoresis. *Acta Histochemica et Cytochemica*.

[4] Bartsch H., Arndt C., Koristka S., Cartellieri M., Bachmann M. (2012). Silver staining techniques of polyacrylamide gels Protein Electrophoresis. *Protein Electrophoresis*.

[5] Berson G. (1983). Silver staining of proteins in polyacrylamide gels: increased sensitivity by a blue toning. *Analytical Biochemistry*.

[6] Merril C. R., Pratt M. E. (1986). A silver stain for the rapid quantitative detection of proteins or nucleic acids on membranes or thin layer plates. *Analytical Biochemistry*.

[7] Nielsen B. L., Brown L. R. (1984). The basis for colored silver-protein complex formation in stained polyacrylamide gels. *Analytical Biochemistry*.

[8] Heukeshoven J., Dernick R. (1985). Simplified method for silver staining of proteins in polyacrylamide gels and the mechanism of silver staining. *Electrophoresis*.

[9] Mirolo L., Schmidt T., Eckhardt S., Meuwly M., Fromm K. M. (2013). pH-dependent coordination of agi ions by histidine: experiment, theory, and a model for sile. *European Journal*.

[10] Allen R. C. (1980). Rapid isoelectric focusing and detection of nanogram amounts of proteins from body tissues and fluids. *Electrophoresis*.

[11] Merril C. R., Goldman D., Sedman S. A., Ebert M. H. (1981). Ultrasensitive stain for proteins in polyacrylamide gels shows regional variation in cerebrospinal fluid proteins. *Science*.

[12] Merril C. R., Dunau M. L., Goldman D. (1981). A rapid sensitive silver stain for polypeptides in polyacrylamide gels. *Analytical Biochemistry*.

[13] de Campos M. R., Botelho A. L., Dos Reis A. C. (2021). Nanostructured silver vanadate decorated with silver particles and their applicability in dental materials: a scope review. *Heliyon*.

[14] Goldberg H. A., Warner K. J. (1997). The staining of acidic proteins on polyacrylamide gels: enhanced sensitivity and stability of "stains-all" staining in combination with silver nitrate. *Analytical Biochemistry*.

[15] Pham N. M., Rusch S., Temiz Y., Beck H.-P., Karlen W., Delamarche E. (2019). Immuno-gold silver staining assays on capillary-driven microfluidics for the detection of malaria antigens. *Biomedical Microdevices*.

[16] Bokhonov B. B., Burleva L. P., Whitcomb D. R., Sahyun M. R. (1998). Electron microscope characterization of AgBr heterojunctions with silver carboxylates and their influence on the morphology of developed silver particles in thermally developed photomaterials. *Microscopy Research and Technique*.

[17] Kumari P., Rickard H., Majewski P. (2012). Deposition of silver and gold nanoparticles on surface engineered silica particles and their potential applications. *Journal of Nanoscience and Nanotechnology*.

[18] Jay G. D., Culp D. J., Jahnke M. R. (1990). Silver staining of extensively glycosylated proteins on sodium dodecyl sulfate-polyacrylamide gels: enhancement by carbohydrate-binding dyes. *Analytical Biochemistry*.

[19] Rabilloud T., Vuillard L., Gilly C., Lawrence J.-J. (1994). Silver-staining of proteins in polyacrylamide gels: a general overview. *Cellular and Molecular Biology*.

[20] Butcher L. A., Tomkins J. K. (1985). A comparison of silver staining methods for detecting proteins in ultrathin polyacrylamide gels on support film after isoelectric focusing. *Analytical Biochemistry*.

